# Factors of Parents-Reported Readiness for Hospital Discharge in Children with Acute Leukemia: A Cross-Sectional Study

This article has been retracted.

**DOI:** 10.1155/2022/4082196

**Published:** 2022-04-22

**Authors:** Wei Cai, Xiaofen Zheng, Runping Wang, Huifen Zhu, Xinxin Xu, Xiaowen Shen, Chunmei Zhang

**Affiliations:** ^1^Department of Cardiology, the Second Affiliated Hospital and Yuying Children's Hospital, Wenzhou Medical University, Wenzhou, 325000, Zhejiang, China; ^2^Department of Pediatric Nephrology, the Second Affiliated Hospital and Yuying Children's Hospital, Wenzhou Medical University, Wenzhou, 325000, Zhejiang, China; ^3^Department of Children's Hematology, the Second Affiliated Hospital and Yuying Children's Hospital, Wenzhou Medical University, Wenzhou, 325000, Zhejiang, China; ^4^Wenzhou Medical University, Wenzhou, 325000, Zhejiang, China; ^5^Department of Nursing, the Second Affiliated Hospital and Yuying Children's Hospital, Wenzhou Medical University, Wenzhou, 325000, Zhejiang, China; ^6^Nursing School, Wenzhou Medical University, Wenzhou, China

## Abstract

**Aim:**

The aim of this study is to investigate the existing status and to explore the influencing factors of parents-reported readiness for hospital discharge in children with acute leukemia (AL) in China and to propose optimizing pathways and recommendations of discharge readiness for clinical reference.

**Methods:**

A cross-sectional survey was conducted for the 122 children with AL who were discharged from the Second Affiliated Hospital and Yuying Children's Hospital, Wenzhou Medical University; their parents were investigated by using the modified Chinese version of Readiness for Hospital Discharge Scale (RHDS) and Quality of Discharge Teaching Scale (QDTS). Data were collected between September 2020 and May 2021.Univariate analysis and multivariate logistic regression analysis were performed to explore the influencing factors of readiness for hospital discharge.

**Results:**

The 122 children with AL included 52 females and 70 males with mean age 6.08 years. The total RHDS score was 7.7 ± 1.2, and 68.9% of the participants had high readiness for hospital discharge (RHDS score >7). The total QDTS score was 7.6 ± 2.0. Parent marital status (OR = 4.86, 95% CI: 1.31–18.05), education status (OR = 3.86, 95% CI: 1.18–12.55), family per capita monthly income (OR = 1.08, 95% CI: 1.01–2.99), and high QDTS (OR = 1.56, 95% CI: 1.11–2.68) were risk factors for high RHDS.

**Conclusions:**

Our data suggest parents of children with AL had high readiness for hospital discharge and had the ability to take care of their children after discharge. Parental marital status, education status, QDTS score, and family per capita monthly income were independently associated with high RHDS.

## 1. Introduction

Acute leukemia (AL) is the most common malignant tumor affecting children [1, 2]. There is approximately 15,000 AL of children in China every year [3]. Adherence to the standard chemotherapy course and timely management of the complications in the course of chemotherapy can increase the initially induced remission rate of childhood acute lymphoblastic leukemia to approximately 95%, the 5-year disease-free survival rate to approximately 80%, and the cure rate to 75%–80% [4, 5]. However, various factors such as multiple hospitalizations, ongoing home care and support, patient follow-up, medical intervention, and long-term medication required during discharge affect treatment efficacy [6, 7]. Parents being the main caregivers of children play a major role in the child's treatment efficacy. The nursing ability of family caregivers of children with AL is inadequate, leading to longer chemotherapy intervals, higher infection rates and unplanned readmissions, higher medical costs, and lower quality of life. Family caregivers of children with AL are affected by many factors, such as the child's treatment stage and treatment duration, caregivers' educational level, care duration, working status, payment mode of medical expenses, family's per capita monthly income, and whether or not a companion helps in child care [8]. Discharge of children with AL can be stressful for caregivers. Therefore, discharge preparation of caregivers is critical, as inadequate discharge preparation can adversely affect post-discharge follow-up needs and outcomes, such as unplanned clinic visits, readmissions, and out-of-hospital deaths [9].

Discharge readiness, first proposed by Fenwick in 1979 [10], refers to an evaluation index for safe discharge by analyzing the ability of patients to leave the hospital, return to society, and further recover based on their physical, psychological, and social health status [11–13]. The evaluation of patients' discharge readiness can effectively prevent the premature discharge of patients, reduce the incidence of post-discharge complications, and reduce the rate of readmission, thus saving medical resources and reducing medical costs [14]. Although the assessment of patient readiness for discharge has been identified as an important part of clinical practice, there has been little research on other factors that can help to improve the readiness of parents with children with AL for discharge. Therefore, this study aimed to assess the associations between readiness for hospital discharge in parents of children with AL; acceptance of disease; and social, demographic, and clinical factors.

## 2. Materials and Methods

### 2.1. Study Design

A cross-sectional survey was conducted for the children with AL who were admitted to the Second Affiliated Hospital of Wenzhou Medical University from September 2020 to May 2021. Inclusion criteria included the following: (a) children (age <16 years) diagnosed with AL according to the International Classification of Diseases-9; (b) parents who had consistent previous care duration ≥2 weeks, at least 6 h a day, and assumed the main role of caregivers of the children after discharge; (c) had no mental disease; and (d) informed consent and voluntary participation in the study. The exclusion criteria were the following: (a) those also diagnosed with severe mental illnesses; (b) decided to leave the hospitals without following medical advice; or (c) refused to participate in the study.

The study was approved by the Ethics Committee of the Second Affiliated Hospital of Wenzhou Medical University (number: LCKY2020-350).

### 2.2. Data Collection

Between September 2020 and May 2021, researchers identified eligible parents of children with AL by reviewing medical records, then asked potential participants about their willingness to participate in the survey. After informed consent was obtained, participants were required to fill out the questionnaires within 4h before discharge. Researchers were trained to adopt a unified guidance language to explain the purpose, significance, and filling methods of the survey to participates. If the participants were diagnosed with dyslexia or visual impairment, the researchers were asked item by item and recorded the choice. The completed questionnaires were collected on the spot. A total of 122 questionnaires were distributed and 122 were effectively received with an effective recovery rate of 100%.

The data of children with AL, including sex, age, pediatric nutritional risk screening score, duration of AL, treatment stage, number of chemotherapies, AL classification, and LOS of hospital, were collected. The general information of parents of children with AL, including age, marital status, number of children, occupation, educational status, income, payment method, and co-caregivers, was gathered.

### 2.3. Readiness for Hospital Discharge Scale and Quality of Discharge Teaching Scale

The RHDS was compiled by Weiss, and it was translated and culturally adjusted by Chen et al. in 2017 [15]. It consists of 22 items, including knowledge (nine items), physical and emotional state (three items for children and four items for parents), expectation support (four items), and pain state (one item for children and parents). Knowledge represents the caregiving ability of parents after discharge. The physical and emotional state describes the physical and emotional readiness of the children and their parents before discharge. Expected support refers to the degree of family social support available after hospitalization. The degree of preparation for the physical comfort of both the child and parent before discharge is indicated by the pain state. The scale is a self-rated summative scale. The first two items are right and wrong questions, which are excluded from the total score. The other 22 items are scored using a 0–10 Likert-type scale, with 0–10 indicating ‘not at all', ‘absolutely', and ‘very much'. Discharge assessment is recommended to be completed within 4h before discharge. The RHDS score ≥7 was high RHDS. Cronbach's *α* was 0.91.

The Quality of Discharge Teaching Scale (QDTS) [16] measures parent perception of the quality of discharge teaching. Recognizing that parents and children receive care from multiple nurses and that discharge teaching occurs throughout the hospitalization, the 18-item QDTS tool asks the parent at the end of the hospitalization to rate the quality of teaching provided by the child's nurses on two subscales [17]. Cronbach's *α* was 0.82.

### 2.4. Statistical Analysis

Stata Statistical Software 16 (Stata Corp LLC) was used for data analysis. All *p*-values were two-sided, and *P-*values <0.05 were considered statistically significant. Continuous data were expressed as mean ± standard deviation (SD), and categorical variables were expressed as frequency. Differences in baseline characteristics in the high RHDS group and low RHDS group were compared via an independent sample *t*-test in continuous variables and *χ*^2^ tests, in categoric variables. Univariate and multivariate logistic regression analyses were used to determine the important variables. Multivariate logistic regression analysis was performed to assess the association between variables and RHDS. Odds ratio (OR) and 95% confidence intervals (CI) were calculated.

## 3. Results

### 3.1. Subject Characteristics

We identified 122 parents of children with AL who met our inclusion criteria. The eligible children with AL included 52 females and 70 males with a mean age of 6.08 years. The number of participants who had low RHDS was 38 (RHDS score< 7). Baseline characteristics are shown in Table 1. Parents in high level of the RHDS group had high levels of married, Medicare payments, higher level of education status, other co-caregivers, number of caregivers, family per capita monthly income, and QDTS score as compared to those in the low RHDS group (*p* < 0.05). The distribution of others did not differ.

### 3.2. Readiness for Hospital Discharge Scale Score and Quality of Discharge Teaching Scale Score

Scores of RHDS are shown in Table 2. The total RHDS score was 7.7 ± 1.2. Regarding the RHDS dimensions, high RHDS groups has higher knowledge (8.9 ± 0.9), physical-emotional status (9.6 ± 0.7), expected support (8.0 ± 2.3), and pain status (9.9 ± 0.5) scores than those of the parents with a low RHDS score.

Scores of QDTS are shown in Table 3. The total score of QDTS was 7.6 ± 2.0. In terms of the quality score of parents' discharge guidance, the content needed before discharge (6.8 ± 2.3), the content actually obtained (7.2 ± 2.5), and the guidance skills and effects (8.0 ± 1.7) were obtained. Regarding the QDTS dimensions, high RHDS groups had higher content needed, content received, and delivery scores than those of the parents with a low RHDS score.

### 3.3. Factors Associated with RHDS

The factors associated with RHDS are shown in Table 4. In univariate analysis, the parent marital status, education status, provider payments, family per capita monthly income, QDTS score, other co-caregivers, and number of caregivers were significantly different (*p* < 0.05). In multivariable analysis, the parent marital status (married) was independently associated with high RHDS (OR = 4.86, 95% CI: 1.31–18.05), parent education status (above high school) was an independent risk factor for high RHDS (OR = 3.86, 95% CI: 1.18–12.55), family per capita monthly income (≥5000) was independently associated with high RHDS (OR = 1.08, 95% CI: 1.01–2.99), and high QDTS was an independent risk factor for high RHDS (OR = 1.56, 95% CI: 1.11–2.68).

## 4. Discussion

### 4.1. Readiness for Hospital Discharge in Parents for Children with AL Was High

In this study, the average score for items of the RHDS was 7.7 ± 1.2, readiness for hospital discharge in parents for children with AL was high, but was not at a satisfactory level, which is lower than that of parental preparation for a child's discharge from the hospital in the United States (8.74 ± 0.97) [18], and also lower than that of parents of hospitalized children with solid organ transplantation (8.6 ± 0.7) [19].This may be due to the different setting of the study investigation. In this study, 68.9% of the participants had high readiness for hospital discharge (RHDS score>7), the average score of the readiness for these participants was 8.5 ± 0.6. We found that most of the parents of children with AL have a good ability to prepare for discharge. This may be due to the long course of disease in children with AL, their parents need to master certain care ability to take care of them during hospitalization, so most parents got ready for hospital discharge.

### 4.2. Influencing Factors Related to the RHDS Score of the Parents of Children with AL

According to the logistic regression analyses, parent marital status, education status, family per capita monthly income, and the total score of the QDTS were independently associated with high RHDS.

#### 4.2.1. Parent Marital Status (Married) and Education Status (above High School) Were Independently Associated with High RHDS of the Parents of Children with AL

Parents' marital status and education status were independently associated with high RHDS. The education level of parents is one of the influencing factors of their discharge care ability. The higher the educational level of the parents, the higher the score of discharge care ability of the parents [20].

Parents' different cultural background, consciousness, concept, under the same conditions, the high education level of parents, in addition to active communication with medical staff exchanges, accepting the medical guidance, receiving care professional knowledge and skills, independently obtaining knowledge in other ways, such as network books, communication with related experience parents, actively listening to other people's guidance, these can be conducive to the improvement of their discharge care ability. The marital status of parents is another influencing factor of their discharge care ability. When the parents were divorced, the child's parents may reduce the time to take care of the child [21], and one person who takes care of a child for a long time may have greater pressure [22].

#### 4.2.2. Family per Capita Monthly Income Were Independently Associated with High RHDS of the Parents of Children with AL

Family per capita monthly income was an independently associated with high RHDS. Smith et al. [23]. showed that the children's annual family income had a statistically significant difference in discharge readiness scores. Lee et al.^22^ showed that low household income was associated with the low health-related quality level of the family. It suggests that financial burden is an important factor influencing family discharge readiness [24, 25].This suggests that higher family income is a protective factor of discharge readiness and provides financial security for the treatment and later recovery of children. In clinical nursing practice, attention should be paid to the overall needs of low-income children's families [26].

In this study, the expected support score of parents in high RHDS group was significantly higher than that in the low RHDS group. Children discharged from hospital often bear the burden of great economic pressure, and the social support resources and coping ability available after discharge are insufficient. Good social support is beneficial for parents of children with AL to better adapt to difficulties and improve their quality of life [27, 28]. Therefore, the social security system of children with AL and their families should be constantly improved, and society should be considerate toward the parents of children with AL [29]. Adequate humanistic care, financial support, and emotional support to reduce their economic and life pressure should be considered by medical and government personnel.

#### 4.2.3. High QDTS Also Was Independently Associated with High RHDS of the Parents of Children with AL

High QDTS was independently associated with high RHDS of the parents of children with AL. Moreover, the knowledge score of parents in high RHDS group was significantly higher than that in low RHDS group [30]. Both of the abovementioned findings suggested that we should do a good job of discharge teaching and it is conducive to improving the score of RHDS [13, 31, 32]. This study encourages nurses to assess RHDS in parents of children with AL at discharge, find the contents that the parents' need, and focus on the contents to strengthen their knowledge. Besides this, the contents that the parents need can be divided into sections, each section could be provided at a time, and retelling and asking questions could be used to confirm that the patients mastered the content. In addition, psychological counseling and health guidance for children, including professional psychological intervention measures to enhance children's resilience should be recommended [33, 34].

This study had some limitations. First the participant of this study included those who AL patient only in 1 hospital in 1 region of Wenzhou, and the results may not be generalized to the whole country. Second, the sample size of 122 is relatively low, which may affect the reliability of the results. Besides that, among 122 parents, only 31 have college education or above, which may not be exactly applied to a patient population with the higher proportion of patients who have college education. Furthermore, a multicenter, large-sample research is necessary prior to widespread conclusion.

## 5. Conclusion

Our data suggest parents of children with AL had high readiness for hospital discharge and had ability to take care of their children after discharge. Parental marital status, education status, QDTS score, and family per capita monthly income were independently associated with high RHDS.

## Figures and Tables

**Table 1:** Characteristics of the patients with acute leukemia.

Characteristic	Low RHDS	High RHDS	*P*
N	38	84	
Child age (years)	6.8 ± 4.2	5.7 ± 3.5	0.132
Child sex (%)			0.476
Male	20 (52.6)	50 (59.5)	
Female	18 (47.4)	34 (40.5)	
Pediatric nutritional risk screening score	2.2 ± 0.6	2.2 ± 0.6	0.147
Duration of AL	8.3 ± 9.4	7.4 ± 8.3	0.264
Treatment stage (%)			0.735
Early induction period	14 (36.8)	36 (42.9)	
Consolidation period	13 (34.2)	22 (26.2)	
Maintenance period	11 (28.9)	25 (29.8)	
Recurrence of treatment	0 (0.0)	1 (1.2)	
Number of chemotherapies	7.8 ± 9.4	7.1 ± 8.4	0.452
AL classification (%)			0.151
ALL	35 (92.1)	69 (82.1)	
AML	3 (7.9)	15 (17.9)	
LOS of hospital	27.9 ± 24.2	21.7 ± 16.7	0.274
Parent/caregiver age (years)	36.4 ± 5.0	34.7 ± 5.6	0.103
Parent marital status (%)			0.001
Married	28 (73.7)	80 (95.2)	
Single	2 (5.3)	0 (0.0)	
Separated/divorced	8 (21.1)	4 (4.8)	
Number of children (%)			0.150
1 child	9 (23.7)	31 (36.9)	
≥2 children	29 (76.3)	53 (63.1)	
Parent education status (%)			0.025
Primary school	28 (73.7)	40 (47.6)	
High school	5 (13.2)	18 (21.4)	
Above	5 (13.2)	26 (31.0)	
Provider payments (%)			0.025
Self-paying	15 (39.5)	17 (20.2)	
Medicare payments	23 (60.5)	67 (79.8)	
Parent employment status (%)		0.093	
Employed	9 (23.7)	33 (39.3)	
Unemployed	29 (76.3)	51 (60.7)	
Other co-caregivers (%)			0.008
No	10 (26.3)	7 (8.3)	
Yes	28 (73.7)	77 (91.7)	
Number of caregivers	1.0 ± 0.9	1.6 ± 1.0	0.002
Monthly income (yuan)			0.049
<5000	35 (92.1)	64 (76.1)	
≥5000	3 (7.9)	20 (23.8)	
QDTS	6.2 ± 0.9	8.1 ± 0.6	0.018

Abbreviations: ALL : Acute Lymphocytic Leukemia; AML : Acute Myelocytic Leukemia; RHDS : Readiness for Hospital Discharge Scale; and QDTS : Quality of Discharge Teaching Scale.

**Table 2:** Results of the RHDS.

RHDS	All	Low RHDS	High RHDS	*P*
Knowledge	8.1 ± 1.6	6.4 ± 1.4	8.9 ± 0.9	<0.001
Physical-emotional status	9.0 ± 1.6	7.6 ± 2.0	9.6 ± 0.7	<0.001
Expected support	7.2 ± 2.7	5.3 ± 2.7	8.0 ± 2.3	<0.001
Pain status	9.1 ± 2.3	7.5 ± 3.5	9.9 ± 0.5	<0.001
Total	7.7 ± 1.2	6.2 ± 0.7	8.5 ± 0.6	<0.001

**Table 3:** Results of the QDTS.

QDTS	All	Low RHDS	High RHDS	*P*
Content needed	6.8 ± 2.3	6.2 ± 1.3	7.1 ± 0.9	<0.001
Content received	7.2 ± 2.5	7.1 ± 2.0	8.0 ± 0.2	<0.001
Delivery	8.0 ± 1.7	6.4 ± 2.5	8.5 ± 2.1	<0.001
Total	7.6 ± 2.0	6.2 ± 0.9	8.1 ± 0.6	<0.001

**Table 4:** Logistic regression of the factors affecting discharge readiness in patients with AL.

Characteristic	Univariable	*P*	Multivariable	*P*
	Or (95% CI)		Or (95% CI)	
Child age (years)	0.93 (0.84, 1.02)	0.1338		
Child sex (%)				
Male	1.0			
Female	0.76 (0.35, 1.63)	0.4764		
Pediatric nutritional risk screening score	1.36 (0.76, 2.41)	0.2970		
Duration of AL	0.99 (0.95, 1.03)	0.5949		
Treatment stage				
Early induction period	1.0			
Consolidation period	0.66 (0.26, 1.66)	0.3741		
Maintenance period	0.88 (0.35, 2.26)	0.7969		
Number of chemotherapies	0.99 (0.95, 1.03)	0.6742		
AL classification				
ALL	1.0			
AML	2.54 (0.69, 9.35)	0.1621		
LOS of hospital	0.98 (0.96, 1.00)	0.1090		
Parent/caregiver age	0.94 (0.88, 1.01)	0.1051		
Parent marital status				
Single/separated/divorced	1.0		1.0	
Married	5.71 (1.60, 20.45)	0.1090	4.86 (1.31, 18.05)	0.0196
Number of children				
1 child	1.0			
≥2 children	0.53 (0.22, 1.27)	0.1530		
Parent education status				
Primary school	1.0		1.0	
High school	2.52 (0.84, 7.59)	0.1003	2.36 (1.76, 7.36)	0.0091
Above	3.64 (1.25, 10.63)	0.0182	3.86 (1.18, 12.55)	0.0123
Provider payments				
Self-paying	1.0		1.0	
Medicare payments	2.57 (1.11, 5.96)	0.0277	2.18 (0.88, 5.42)	0.1156
Parent employment status				
Employed	1.0			
Unemployed	0.48 (0.20, 1.14)	0.0966		
Other co-caregivers				
No	1.0		1.0	
Yes	3.93 (1.36, 11.32)	0.0113	2.40 (0.72, 8.04)	0.3082
Number of caregivers	1.99 (1.21, 3.27)	0.0069	1.54 (0.35, 6.67)	0.5661
Monthly income (yuan)				
<5000	1.0		1.0	
≥5000	1.48 (1.20, 1.94)	0.0023	1.08 (1.01, 2.99)	0.0019
QDTS	3.41 (2.19, 5.03)	0.0019	1.56 (1.11, 2.68)	0.0011

## Data Availability

The data used and/or analyzed during the current study are available from the corresponding author (Chunmei Zhang) on reasonable request.
